# The Addition of ROTEM Parameter Did Not Significantly Improve the Massive Transfusion Prediction in Severe Trauma Patients

**DOI:** 10.1155/2022/7219812

**Published:** 2022-10-15

**Authors:** Dongyup Baik, Seok-Ran Yeom, Sung-Wook Park, Youngmo Cho, Wook Tae Yang, Hoon Kwon, Jae Il Lee, Jun-Kyeung Ko, Hyuk Jin Choi, Up Huh, Tae Sik Goh, Chan-Hee Song, Lee Hwangbo, Il Jae Wang

**Affiliations:** ^1^Department of Emergency Medicine, School of Medicine, Pusan National University and Biomedical Research Institute, Pusan National University Hospital, Busan 49241, Republic of Korea; ^2^Department of Radiology, Biomedical Research Institute, Pusan National University Department of Radiology, Busan 49241, Republic of Korea; ^3^Department of Neurosurgery, Biomedical Research Institute, Pusan National University Hospital, Busan 49241, Republic of Korea; ^4^Department of Thoracic and Cardiovascular Surgery, School of Medicine, Pusan National University, and Biomedical Research Institute, Pusan National University Hospital, Busan 49241, Republic of Korea; ^5^Department of Orthopaedic Surgery, Biomedical Research Institute, Busan National University Hospital, Busan National University School of Medicine, Busan 49241, Republic of Korea; ^6^Department of Biomedical Engineering, Graduate School, Pusan National University, Busan 49241, Republic of Korea

## Abstract

**Background:**

Rotational thrombelastometry (ROTEM) has been used to evaluate the coagulation state, predict transfusion, and optimize hemostatic management in trauma patients. However, there were limited studies on whether the prediction value could be improved by adding the ROTEM parameter to the prediction model for in-hospital mortality and massive transfusion (MT) in trauma patients.

**Objective:**

This study assessed whether ROTEM data could improve the MT prediction model.

**Method:**

This was a single-center, retrospective study. Patients who presented to the trauma center and underwent ROTEM between 2016 and 2020 were included. The primary and secondary outcomes were massive transfusions and in-hospital mortality, respectively. We constructed two models using multivariate logistic regression with backward conditional stepwise elimination (Model 1: without the ROTEM parameter and Model 2: with the ROTEM parameter). The area under the receiver operating characteristic curve (AUROC) was calculated to assess the predictive ability of the models.

**Result:**

In total, 969 patients were included; 196 (20.2%) received MT. The in-hospital mortality rate was 14.1%. For MT, the AUROC was 0.854 (95% confidence interval [CI], 0.825–0.883) and 0.860 (95% CI, 0.832–0.888) for Model 1 and 2, respectively. For in-hospital mortality, the AUROC was 0.886 (95% CI, 0.857–0.915) and 0.889 (95% CI, 0.861–0.918) for models 1 and 2, respectively. The AUROC values for models 1 and 2 were not statistically different for either MT or in-hospital mortality.

**Conclusion:**

We found that the addition of the ROTEM parameter did not significantly improve the predictive power of MT and in-hospital mortality in trauma patients.

## 1. Introduction

A preprint has previously been published [1]. Traumatic hemorrhage is a major cause of mortality and a significant preventable cause of death. Nearly 50% of deaths within 24 hours of trauma are caused by uncontrolled hemorrhage, and most hemorrhage patients die within 2 hours of presenting to the hospital [2]. In addition, massive traumatic bleeding could induce trauma-induced coagulopathy, which is associated with higher morbidity and mortality rates 3–6. Many strategies have been developed to improve outcomes for patients with severe bleeding, including an early balanced transfusion, permissive hypotension, limited crystalloids, and a massive transfusion protocol (MTP) [3–6]. Previous studies have shown that using MTP can improve patient prognosis, and many trauma centers have implemented MTP [4, 5, 7, 8].

Several tools have been introduced to identify patients requiring massive transfusion (MT) and to accurately activate the MTP. These tools include physiologic variables such as altered mentality, tachycardia, hypotension, and laboratory variables such as hemoglobin and base excess [9]. Furthermore, to predict MT more accurately, scoring systems in which various variables are combined have been developed; these scoring systems include trauma-associated severe hemorrhage (TASH), ABC, Prince of Wales Hospital, and traumatic bleeding severity scores [10–12]. However, it is still challenging to identify which patients will require MT.

Recently, there has been an increased use of viscoelastic hemostatic assays (VHA), such as thromboelastography (TEG) and rotational thromboelastometry (ROTEM), for trauma patients [13, 14]. Compared to conventional coagulation tests, VHA provides a whole coagulation cascade from the initiation of clot formation to the breakdown of the clot in real time [15, 16]. As it can measure the lysis state, which is impossible with a conventional coagulation test, VHA can diagnose the pathological lysis state, such as hyperfibrinolysis and fibrinolysis shutdown [17–21]. Previous studies have assessed the predictive value of VHA for trauma and identified the VHA parameter as a valuable predictor of mortality, transfusion, and coagulopathy in trauma patients [21–26]. However, no studies have been conducted on the added value of VHA data in predicting trauma outcomes compared with prediction models without VHA data.

This study aimed to assess whether ROTEM data could improve the MT prediction model. We hypothesized that ROTEM data could enhance the value of the MT prediction model.

## 2. Materials and Methods

### 2.1. Study Design and Setting

This retrospective, single-center study was conducted at the trauma center of a 1400-bed, university-affiliated hospital in Busan, South Korea. Our trauma center is a level I regional trauma center that is responsible for approximately 7 million people. It is one of the largest trauma centers in South Korea, and almost 1,000 trauma patients with an injury severity score (ISS) > 15 are managed annually. This study was approved by the Institutional Review Board of our hospital (2208-014-118). Informed consent was waived because the data were analyzed anonymously and retrospectively. The study was conducted in accordance with the tenets of the Declaration of Helsinki.

#### 2.1.1. Study Population

Consecutive patients who presented to the trauma center between 2016 and 2020 and underwent ROTEM were included. Patients under the age of 15 years, those with pre-hospital cardiac arrest, and those with missing values were excluded.

### 2.2. Data and Outcome Variables

Data were obtained from the hospital trauma registry and electronic medical records. Data included age, sex, and the following laboratory data were collected at the emergency department (ED) presentation: vital signs (systolic blood pressure [SBP] and heart rate [HR]), Glasgow coma scale (GCS) score, prothrombin time international normalized ratio (PT INR), activated partial thromboplastin time (aPTT), hemoglobin level, platelet count, and ROTEM data. Furthermore, data included packed red blood cells (PRBC) transfused within the first 24 h, ISS, 24-hour mortality, and in-hospital mortality.

We performed the VHA test using the ROTEM delta (TEM International GmbH, Munich, Germany). Based on the mechanism of injury, hemodynamic status, and focused assessment with sonography in trauma (FAST) results, the physician decided whether to perform the ROTEM test. We collected the EXTEM clotting time (CT), maximum clot firmness (MCF), and maximum lysis (ML). Our primary outcome was MT, whereas the secondary outcome was in-hospital mortality. We defined MT as the transfusion of more than 10 units of packed red blood cells within 24 h [5].

### 2.3. Statistical Analysis

Continuous variables were described as the mean ± standard deviation, while categorical variables were described as numbers (percentages). Baseline demographic and clinical data were compared using either Student's t-test for continuous variables or the Chi-square test for binomial variables. We chose stepwise logistic regression analyses with backward elimination for primary and secondary outcomes. The receiver operating characteristic (ROC) curve of the regression models with or without ROTEM data enabled a visual comparison of the models. Calculating the AUROC allowed the quantitative assessment of the regression models. DeLong's method estimated the 95% confidence interval (CI) for each AUROC. All statistical analyses were performed using R 4.1.3 (R Foundation for Statistical Computing, Vienna, Austria).

## 3. Result

### 3.1. Baseline Characteristics and Comparison of the MT and Non-MT Patients

Initially, 1033 patients met the inclusion criteria between 2016 and 2020. The following patients were excluded: age <15 years (*n* = 10), prehospital cardiac arrest (*n* = 44), and missing values (*n* = 10). A total of 969 patients were included in this study. There were 735 male patients (75.8%) with a mean age of 56. The mean ISS score was 23.6 (11.9–35.3), 196 patients received MT (20.2%), and the in-hospital mortality rate was 14.1%. The characteristics of the study population are summarized in Table 1.

The MT and non-MT groups were compared (Table 2). The SBP (*p* < 0.001), GCS (*p* < 0.001), hemoglobin level (*p* < 0.001), and platelet count (*p* < 0.001) in the MT group were significantly lower than those in the non-MT group. PR (*p* < 0.001), PT (*p* < 0.001), and APTT (*p* < 0.001) were significantly higher in the MT group. We found no significant differences in sex or age between the two groups. The MT group had higher EXTEM CT (*P*=0.019), EXTEM ML (*p* < 0.001), and lower EXTEM MCF (*p* < 0.001) than the non-MT group. The characteristics of the study population are summarized in Table 2.

#### 3.1.1. Logistic Regression and ROC Analysis

We performed stepwise logistic regression analyses with backward elimination for primary and secondary outcomes. The regression model for MT without ROTEM data (Model (1) selected SBP, PR, GCS, hemoglobin, platelets, and PT as predictors. The model with ROTEM data (Model (2) included EXTEM MCF and EXTEM while dropping the platelet count from the former (Table 3). The corresponding AUROC for model 1 was 0.8542 (95% CI, 0.8250–0.8833); and Model 2 was 0.8603 (95% CI, 0.8321–0.8885) (Figure 1). For in-hospital mortality, the AUROC of Model 1 was 0.8864 (95% CI, 0.8575–0.9152) and Model 2 was 0.8899 (95% CI, 0.8618–0.9181) (Figure 2). All primary and secondary outcome models demonstrated statistically insignificant differences between models with and without ROTEM data (*p*=0.085 and *p*=0.566, respectively).

## 4. Discussion

The objective of this study was to evaluate whether the addition of ROTEM data could improve the ability of the prediction model. We constructed two logistic regression models (Model 1: without ROTEM data, Model 2: with ROTEM data) and identified that the added ROTEM data did not significantly improve predictive accuracy. Although EXTEM CT and EXTEM ML were significantly associated with MT and the AUROC of Model 2 was higher than that of Model 1, there was very little difference in AUROC between the two models.

Accurately identifying the needs of MT and activating the MTP is essential in order to lower mortality in severely injured trauma patients with massive bleeding [2, 27–30]. Previous studies have suggested various scoring systems and models for MT prediction. These models used diverse variables, including demographic data, clinical findings, hemodynamic status, injury mechanism, FAST results, and laboratory data [10–12]. Yücel et al. introduced a scoring system called the TASH score. The TASH score utilized seven variables, such as laboratory and physiologic data, including SBP, hemoglobin level, the FAST result, the presence of long bone fracture, HR, base excess, and sex [10]. The ABC scoring system was developed in 2009 and consists of four dichotomous components: the mechanism of injury, the FAST result, SBP, and HR. The ABC scoring system is broadly used because it has the advantage that components of the scoring system can be acquired early in the assessment phase but are as effective as the prior TASH scoring system. The AUROC of the ABC and TASH scores were 0.859 and 0.842, respectively. However, the difference between the two scores was not statistically significant [11].

Two prediction models were constructed. The first model (Model 1) consisted of six variables selected without ROTEM variables by stepwise logistic regression analyses with backward elimination. Then, SBP, HR, GCS score, hemoglobin concentration, platelet count, and PT were chosen. Each selected variable was statistically significant with a *p*value lower than 0.05. The AUROC of the model using these 6 variables was 0.8542. Our model has a predictive value that is similar to that of the previously introduced scoring system.

For the second prediction model (Model 2), we added ROTEM data. Among the various ROTEM variables, EXTEM CT, MCF, and ML were selected. CT is the time from the start of the test until a clot firmness amplitude of 2 mm, and MCF is the maximum amplitude of clot firmness. The CT and MCF are basic and crucial indicators for identifying the initiation of coagulation and the firmness of the clot, respectively. ML indicates maximum lysis during the runtime and is expressed as a percentage of MCF [16]. Among the parameters representing coagulation activation, clot firmness, and clot lysis, we selected the most important variables one by one and added them to the model. MCF and ML were selected through a stepwise backward elimination process, and platelet counts were excluded. The AUROC of the second model, using seven variables, including ROTEM data, was 0.8603. The AUROC of Model 2 showed higher performance, but it was not statistically significant.

In our study, it is unclear why additional ROTEM data did not improve the predictive power. One possible explanation is that, despite ROTEM's unique strengths, the results are correlated with conventional coagulation tests [31, 32]. Haas et al. showed ROTEM's correlation with conventional coagulation tests in pediatric patients, and Schöchl et al. suggested that ROTEM-guided administration of fibrinogen concentrate and prothrombin complex concentrate was fast and effective [33, 34]. We believe that adding the corresponding variable could not provide a major contribution to improving the prediction model.

Another explanation is that our study did not investigate the relationship between the ROTEM parameters. In this study, three variables were thought to represent the crucial points of the coagulation cascade and were chosen to assess the relationship with the needs of the MT. In the ROTEM test, multiple chambers with various parameters are suggested. Further studies must be conducted to delineate the relationship between MT and other ROTEM parameters to improve the prediction model.

Our study had several limitations. First, because this study was retrospective, bias could exist. Second, this was a single-center trauma study. Further validation and multicenter studies are required to generalize the clinical relevance of these findings. Another limitation was that we did not separately classify patients with traumatic brain injury (TBI). Patients with TBI have different characteristics and prognoses. Fourth, the physician decided whether to perform the ROTEM test based on the hemodynamic state, FAST result, and mechanism of injury rather than a protocol. Finally, we use only three ROTEM variables. We considered these variables to be the most important; however, it is possible that the result could be altered if additional ROTEM variables were added.

## 5. Conclusion

In conclusion, our study identified that ROTEM variables were independently related to MT and in-hospital mortality in patients with trauma. However, adding them to the prediction model did not significantly enhance its predictability.

## Figures and Tables

**Figure 1:** ROC analysis for MT.

**Figure 2:** ROC analysis for in-hospital mortality.

**Table 1:** Baseline characteristics. SD: standard deviation; SBP : Systolic blood pressure; GCS : Glasgow coma scale; PT (INR): prothrombin time (international normalized ratio); aPTT: activated partial thromboplastin time; CT: clotting time; MCF: maximum clot firmness; ML: maximum lysis; ISS: injury severity score.

Variable	Total (*n* = 969)
Age (mean ± SD)	56.0 ± 18.0
Sex, *n* (%)	
F	234 (24.2)
M	735 (75.8)
SBP (mean ± SD)	99.8 ± 36.9
Pulse rate (min^−1^) (mean ± SD)	97.1 ± 23.2
GCS (mean ± SD)	11.9 ± 4.3
Hemoglobin (g/dL) (mean ± SD)	12.1 ± 2.5
Platelet (10^3^/*μ*L) (mean ± SD)	212.1 ± 73
PT (INR) (mean ± SD)	1.26 ± 0.78
aPTT (sec) (mean ± SD)	35.3 ± 24.1
EXTEM CT (mean ± SD)	105.8 ± 341.7
ECTEM MCF (mean ± SD)	56.5 ± 12.4
EXTEM ML (mean ± SD)	5.0 ± 21.6
ISS (mean ± SD)	23.6 ± 11.7
Massive transfusion, *n* (%)	
No	196 (20.2)
Yes	773 (79.8)
24-hour mortality, *n* (%)	
No	915 (94.43)
Yes	54 (5.57)
In-hospital mortality, *n* (%)	
No	832 (85.9)
Yes	137 (14.1)

**Table 2:** Comparison of clinical characteristics and outcomes between non-massive transfusion groups and massive transfusion groups. SD: standard deviation; SBP : Systolic blood pressure; GCS : Glasgow coma scale; PT (INR): prothrombin time (international normalized ratio); aPTT: activated partial thromboplastin time; CT: clotting time; MCF: maximum clot firmness; ML: maximum lysis; ISS: injury severity score.

Variable	Non-massive transfusion group (*n* = 773)	Massive transfusion group (*n* = 196)	*P*-value
Age (mean ± SD)	56.3 ± 18.0	54.8 ± 18.0	0.2987
Sex, *n* (%)			0.1804
F	179 (23.2)	55 (28.1)	
M	594 (77.5)	141 (71.9)	
SBP (mean ± SD)	107.3 ± 35.0	70.4 ± 28.7	<0.0001
Pulse rate (min^−1^) (mean ± SD)	95.1 ± 22.8	104.8 ± 23.6	<0.0001
GCS (mean ± SD)	12.6 ± 4.0	9.4 ± 4.9	<0.0001
Hemoglobin (g/dL) (mean ± SD)	12.5 ± 2.3	10.6 ± 2.7	<0.0001
Platelet (10^3^/*μ*L) (mean ± SD)	219.1 ± 70.7	184.6 ± 75.8	<0.0001
PT (INR) (mean ± SD)	1.14 ± 0.41	1.72 ± 1.44	<0.0001
aPTT (sec) (mean ± SD)	30.9 ± 14.8	52.4 ± 40.7	<0.0001
EXTEM CT (mean ± SD)	86.8 ± 264.5	180.6 ± 543.8	0.01991
ECTEM MCF (mean ± SD)	58.5 ± 10.8	48.7 ± 15.3	<0.0001
EXTEM ML (mean ± SD)	7.5 ± 14.3	22.6 ± 36.4	<0.0001
ISS (mean ± SD)	21.6 ± 11.1	31.3 ± 10.6	<0.0001

**Table 3:** Parameter estimates of Logistic Regression for Model 1 containing only Clinical Data, and Model 2 containing Clinical and ROTEM Data, as predictors of Massive Transfusion. SBP : Systolic blood pressure; GCS : Glasgow coma scale; PT (INR): prothrombin time (international normalized ratio); MCF: maximum clot firmness; ML: maximum lysis.

	Model 1			Model 2		
Covariate	Estimate	Standard error	*P*-Value	Estimate	Standard error	*P*-Value
SBP (mmHg)	−0.029498	0.003618	0.00234	−0.027282	0.003653	<0.0001
Pulse rate (min^−1^)	0.010161	0.004005	0.01117	0.010049	0.004015	0.012317
GCS	−0.096050	0.021846	<0.0001	-0.079226	0.022501	0.000430
Hemoglobin (g/dL)	−0.114647	0.043657	0.00864	−0.140123	0.041306	0.000693
PT (INR)	0.505367	0.192942	0.00881	0.401785	0.195082	0.039439
PLT (10^3^/*μ*L)	−0.002741	0.001449	0.05854	—	—	—
EXTEM MCF	—	—	—	−0.018814	0.008288	0.023210
EXTEM ML	—	—	—	0.007221	0.004069	0.075997

## Data Availability

The datasets used and/or analyzed during the current study are available from the corresponding author on reasonable request.
